# A Data-Enabled Business Model for a Smart Healthcare Information Service Platform in the Era of Digital Transformation

**DOI:** 10.1155/2021/5519891

**Published:** 2021-06-01

**Authors:** Yu Su, Fei Hou, Mingde Qi, Wanxuan Li, Ying Ji

**Affiliations:** ^1^Institute of Advanced Studies in Humanities and Social Science, Beijing Normal University, Zhuhai 519087, China; ^2^Management School, Guangdong University of Technology, Guangzhou 510520, China; ^3^School of Business, Dalian University of Technology, Panjin 124221, China

## Abstract

Digital technology has promoted service innovation and provided effective technical support for public service innovation in recent years. Smart healthcare, a key element of smart city development, has gradually become an important issue in government administration. Digital technology is deeply embedded in healthcare services and reshapes value creation through digital transformation. This study combines data-enabled platform business models and value cocreation and adopts a case study approach to develop a business model for a medical information service platform that allows stakeholders to cocreate value through service exchange and resource integration in smart healthcare ecosystems, promotes efficient and coordinated applications of information, and realizes innovative development in the medical industry.

## 1. Introduction

With the trend of “digital + public service” integration, digital technologies that enable public service innovation have gradually become an important issue. As a key element of the smart city design, smart healthcare attempts to connect patients, doctors, hospitals, medical equipment, information systems, and intelligent systems through information and Internet technologies to collect and integrate medical cloud data and form medical cloud data centers, thereby realizing information sharing and interactions among patients, medical workers, medical institutions, and firms in the healthcare industry. An intelligent medical system can thus better serve patients, help hospitals make science-based management decisions, and work toward the goal of smart healthcare [1]. This system is characterized by interconnection, collaboration, and reliability, and it can help address issues commonly seen in the medical system, including high medical costs, inequitable resource allocation, and low efficiency.

Medical service innovation in the context of digital transformation is a cross-departmental and cross-level collaboration involving systematic innovation on the part of government, enterprises, the public, and other participants. Digital technology has stimulated multidimensional boundaryless innovation in technology, management, and institutions. These changes, in turn, have elicited new demands for digital technology and triggered innovative restructuring of organizations, product and service supply modes, and governance policy leading to reallocation of the resources of stakeholders and thereby creating new management modes and rules [2]. Currently, digital innovation models of public services include government-led, government-sponsored (industry-driven), and enterprise-led (provision of platforms). “Government-led” governance does not meet the current complex public healthcare application scenarios. The distributed and decentralized platform governance model has gradually become the new trend in public service innovation.

Based on data-enabled business model theory and service ecosystem theory, and with smart healthcare as an example, this paper develops a medical information service platform business model that integrates the interests of all stakeholders, forms a new ecosystem of healthcare information through value cocreation, and thereby drives the cross-border integration and development of the smart healthcare industry.

## 2. Theory

### 2.1. Public Service Digital Innovation

The essential demand of public service innovation is the digital transformation of the social technology system, and the ultimate goal is to achieve value cocreation. Goods-dominant logic, which is based on the industrial economy and an industrial model, emphasizes the specialization-based division of labor. Therefore, there is a clear boundary between goods and services under this model, and values are embedded in visible goods [3, 4]. In contrast, service-dominant logic provides a theoretical foundation for the intrinsic connection between modern service innovation and value cocreation [5]. Service innovation realizes value cocreation through resource integration and capacity interaction, and interaction is the source of value creation [6].

Smart healthcare is a digital innovation in the public service sector. In contrast to the service and manufacturing sector, public service suppliers are more diversified. The public sector provides a variety of public services through cooperation with other government departments, private enterprises, nongovernmental organizations, communities, and public individuals. The essential demand of public service innovation is the reconstruction of a social framework adapting to technological change.

In the era of digital transformation, digital technology enables the elements of public service innovation and provides opportunities to multiple participants in public service innovation and the possibility of value cocreation [7]. Therefore, the goal of public service innovation is to shift gradually from “service supply” to “value cocreation.”

### 2.2. Data-Enabled Platform Business Model

The development of big data technology enables firms to better cope with the scale and complexity of data, and progress in digital technology has created new business opportunities and changed the ways in which firms create, deliver, and capture value [8]. Big-data-based business model innovation has been recognized by many firms and scholars.

Based on the “digital value chain” concept, the process of gaining economic value from data can be divided into four phases: data collection, data aggregation, data analysis, and data use and monetarization [9]. Business models can be classified as either data-enhanced or data-enabled models depending on the different roles and uses of data in the models. For data-enhanced business models, the digitalization of “incremental business” helps coordinate existing business operations, facilitate decision-making, and improve or create products and services, but the data do not change or determine the core business model. In comparison, data-enabled models are fully digitalized business models that completely rely on data to develop revenue-generating strategies. For this type of business model, massive amounts of data and advanced data analytics capabilities are the key factors of production for the core revenue-generating activities of the firm. Firms employing this type of business model mainly include online platforms that rely on selling data or providing data analytics services.

The development of digital technology has promoted the emergence of a large number of platform-based firms, and platforms have become a medium that connects firms, suppliers, distributors, and customers [10]. The platform business model connects and integrates multiple groups and thereby reduces the transaction cost of each stakeholder and capitalizes on the network effect. With the development of digital technology, the establishment of a platform-based business model to enable the gradual transition from value creation to value cocreation has become the focus of studies on business model innovation [11–13].

Public service providers are more diversified than firms in other service sectors. Public value is created not only by the public sector alone, but also by the common responsibility of the government, citizens, enterprises and other social organizations. The platform business model provides a new approach and perspective for public service innovation to coordinate the cooperation of multiple departments and various participants.

### 2.3. Value Cocreation from the Perspective of Service Ecosystems

Value cocreation originated from coproduction, in which firms allow customers to participate in production and service provision, and value is cocreated through interactions among participants. Big data and Internet technologies have enabled products and services that are digitalized and intellectualized, thereby reshaping industry competition and industry boundaries and transforming the mechanisms of value creation interaction [14].

Since the development of the Internet economy, value cocreation has focused on the network relationship, in which multiple players create value together, and suppliers, business partners, collaborators, and customers cocreate value [15] within a service ecosystem. The service ecosystem takes a macroscopic perspective by viewing all socioeconomic players as important components of value creation [16].

From the service ecosystem perspective, value cocreation incorporates the participants of socioeconomic activities into the value cocreation process, views institutions and intensive interactions as the core of value cocreation, and realizes value cocreation by integrating socioeconomic resources and service exchange [17]. The service ecosystem under value cocreation emphasizes user participation and the important roles that user resources play in the value creation network, as well as the ability of platforms to activate the user network effect and thereby transform platform users from passive value recipients to active value developers and creators.

### 2.4. Sustainable Platform Business Model

The platform is one of the most significant business model innovations of value cocreation [18]. Driven by interests, the platform business model innovation process may appear to sacrifice the long-term interests of users for value orientation, which reduces the trust of consumers and affects the sustainability of the platform business model. Therefore, the switch from a platform business model to a sustainable platform business model has become a prominent topic.

A sustainable business model is defined as a tool that integrates sustainability into a company's value proposition and value creation logic [19]. The sustainable platform business model incorporates sustainability and social responsibility into the platform business model. Furthermore, it integrates environmental, social, and economic value at the value proposition level and, at the value distribution level, allows residual value to be shared by the participants of the entire platform business ecosphere and the social ecosphere, in which the platform is embedded, thereby creating shared value that covers the economy, society, and the environment [20, 21].

## 3. Development of a Data-Enabled Business Model for a Smart Healthcare Information Service Platform

### 3.1. Theoretical Framework

In the big data era, data are transparent, and their economic value is amplified. Furthermore, data lead to the reallocation of resources, resulting in new management models and rules. This study developed a framework based on the customer service platform and the data-enabled business model, as shown in Figures 1 and 2.

This framework explains the design principle of the data-enabled business model of information service platforms; it is an information sharing and interaction model, with a focus on the information platform, and it is based on the data-enabled business model and the customer service platform business model. Equipped with advanced technologies such as artificial intelligence, the Internet of Medical Things (IoMT), wireless sensors, data cloud computing, and big data, the information service platform collects, stores, transforms, organizes, and transmits medical data. In particular, based on the needs of cloud computing, the platform transforms and analyzes data to scientifically integrate various types of data resources and then provides the processed data to stakeholders of the platform.

### 3.2. Research Design

#### 3.2.1. Method Selection

In view of the lack of academic research on smart healthcare service platforms, more information needs to be collected. The case study approach was adopted for this research. A case study is both a qualitative method that can be used to analyze the attributes of the research object and draw conclusions and an empirical method that can be used to study phenomena. The case study method can be used to clarify internal business rules and management logic and thereby improve the design of a business model.

#### 3.2.2. Case Selection

The development of a smart healthcare service system needs to be oriented toward patients, healthcare professionals, medical institutions, and health regulatory and supervisory agencies. The business model of the smart healthcare service platform aims to promote the transformation of traditional relationships in healthcare service systems with the development and application of information technology and form a healthy ecosystem through the industrial aggregation function of the smart medical information service platform. The smart healthcare ecosystem, which is formed via multidisciplinary and cross-industry integration, involves many stakeholders, including consumers, policy makers and regulators, technology providers, service providers, medical service payers, and capital investors.

This case study aims to investigate the potential participants of the intelligent medical service platform and understand their needs and value proposition, improve the ability of the platform model to meet the needs of stakeholders, and enhance value cocreation. Accordingly, eight institutions in the Pearl River Delta area in Guangdong Province, China, including two hospitals and six stakeholders, were selected for the survey in this study. To ensure the reliability of the information in the case study, the availability of information and the industrial characteristics and representativeness of the institutions were considered when selecting the interview samples.

#### 3.2.3. Data Collection

To ensure that the design of the platform business model was reasonable, the stakeholders of the smart healthcare information service platform were interviewed. For the institutions interviewed, we collected first-hand data through field research and semistructured interviews, and after the interviews, we verified and supplemented the data through online channels such as emails and phone calls; in addition, second-hand data were obtained for quantitative analysis and verification. The data sources for the stakeholders in this case study are shown in Table 1.

#### 3.2.4. Conclusion of the Analysis

The stakeholders and their interests in the smart healthcare ecosystem were summarized based on the interviews and the related research, as shown in Table 2, to provide a basis for the design of the business model for the smart healthcare information service platform.

The users of the smart healthcare system are the consumers who receive healthcare services. Their role in the ecosystem is to guide demand. Personalized user needs are the basis of decisions on policy, technology, service, payment, and investment. The supervisor in the smart healthcare system refers to the government's policymaking and supervisory departments, which incentivize and regulate policies for the smart healthcare system and the healthy development of the industry by providing legal protection for various stakeholders and helping all parties actively enter the smart healthcare system.

Professional healthcare service providers, as represented by large general hospitals, private hospitals, and physical medical examination centers, are all aware of the impact of big data on the traditional medical industry and are actively participating in the construction of the smart healthcare ecosystem. They are willing to cooperate with other stakeholders to improve the use of medical resources and the quality of healthcare by digitizing and scientifically managing the internal information (e.g., pharmaceuticals, personnel, and equipment) of healthcare service providers. With the continuous improvement in big data and data mining technology, computer-aided systems can be used to improve the efficiency and accuracy of medical treatment by examining the relationship between patients and diseases. Medical R&D institutions, as represented by research institutes and pharmaceutical firms, are actively exploring ways to use medical big data, including patient access information, clinical medical research and laboratory data, and health management information generated by smart wearable devices, for R&D applications. By acquiring integrated demand information based on healthcare activities, the suppliers of medical products and services provide personalized products and services based on the demands of interest groups. Active participation in the capital market is also indispensable to the development of the smart healthcare ecosystem, with various investment partners jointly participating in the construction of the smart healthcare system to explore potential market opportunities.

In an ideal smart healthcare ecosystem, stakeholders need to adjust their roles and contribute resources such as technology, services, and funds to the system. In the new ecosystem, the interests of stakeholders should be mutually supportive.

### 3.3. Smart Healthcare Information Service Platform

#### 3.3.1. Data Integration

Data are key to production in the data-enabled business model. The data available in the smart healthcare system are classified into two categories: hospital management data and patient data. Big data technologies enable centralized management and the sharing of all types of data in the medical system (e.g., medical imaging data such as computed tomography (CT), B-scan, and magnetic resonance imaging (MRI) data as well as diagnosis, treatment, and medication data). Patient data mainly include basic medical data (e.g., wearable device data such as temperature, blood pressure, heart rate, and other real-time patient data); medical examination results, which can be transferred from the built-in IoMT modules of medical equipment for the screening, diagnosis and treatment of diseases; and long-term monitoring data such as blood glucose data, which can be used to provide early warnings for diabetes and adjust medications. These data need to be stored and used with special attention to information privacy and security.

In addition to technology implementation, the experience of the users of public services should be considered. Most of the previous studies have focused on the technical feasibility of smart healthcare while neglecting the psychological needs of users. The functions of the smart healthcare system are usually restricted by their ability to satisfy the psychological needs of users. With continuous improvement in meeting personalized demand, mining and integrating information on platform user demand to improve user satisfaction will greatly improve healthcare products and services.

#### 3.3.2. Platform Modularization

Modularity, as a prominent feature of platform organization, plays a key role in the establishment and governance of platforms [22]. From the perspective of organizational design, through modular architecture and configuration, a platform dynamically coordinates partners with different resources and different businesses and improves operational efficiency [23].

By analyzing stakeholders in the healthcare industry, the unique modular system of the platform was designed to coordinate the ecology of participants to adapt to the diversified and changing needs of platform users. The platform was divided into three main modules, i.e., product, service, and information, as shown in Figure 3. By providing services to individuals, families, communities, hospitals, etc. and connecting and interacting with government, social security, pension institutions, and other partners, the platform captures market demand information, aggregates and processes the information, shares information with stakeholders, encourages platform participants to improve products and services, and enhances diversity among modules.

#### 3.3.3. Platform Governance

The platform model breaks the traditional organizational management structure and integrates participants at different levels or in different fields. There is no obvious boundary or supervision, and collaborative governance is the key to the success of the platform model. The essence of collaborative governance is a new model of governance under the guidance of cooperation, which emphasizes open and rational dialogue, exchange and consultation among government, corporations, and society on the basis of equality to develop and maintain deep mutual trust and understanding and to form a dynamic balance among stakeholders [24, 25]. A smart healthcare service platform implies decentralized collaborative governance. As the service initiator, the government takes the lead in proposing application requirements, establishing a special working group composed of government departments and enterprise research and development (R & D) teams, and issuing relevant policies. Hospitals, enterprises and social organizations are important participants, forming a beneficial collaborative and interactive ecology. Finally, the platform application is promoted by the community and other grassroots organizations, and the public can obtain the required services and data and play a supervisory role.

In the digital economy era, the platform coordinates the distributed ecosystem of participants through modular architecture and manages the platform modules through the openness of the platform. The platform may set the openness level based on the modules' characteristics, but in general, it is characterized by a high degree of participation and low transparency. A high degree of participation eases the restrictions imposed on external organizations and individuals and attracts complementors to improve the platform's products and services and thereby realize value creation, while low transparency limits excessive information exchange and thereby retains the core factors of production, including private medical information, within the platform.

#### 3.3.4. Platform Ecosystem

The boundary of the ecosystem can be changed and expanded to foster business model innovation. Cross-border integration is an inevitable development in the healthcare industry. The model of the smart healthcare information service platform incorporates the interests of stakeholders into its design to build a cross-border integrated ecosystem [11]. As a new cross-border integrated ecosystem, smart healthcare involves a number of multidisciplinary, cross-sector stakeholders, including users, policymakers, supervisors, R&D institutions, technology and service suppliers, and capital markets, who coexist within the dependency model of resource complementarity. The platform business model coordinates the distributed ecosystem of participants through its modular architecture to promote resource circulation and allocation, as shown in Figure 4. In addition, it controls and manages its modules by using openness to enhance the diversity and interdependence of various parts of the ecosystem.

Traditional platform business models mainly focus on a rapid increase in commercial value (i.e., economic value); however, sustainable platforms also emphasize social and environmental value. Unlike that of other business service platforms, the value proposition of a healthcare platform must be oriented toward comprehensive economic, social, and environmental value that aims to improve the efficiency of allocation of healthcare resources in society and to effectively manage and control interactions and transactions, various types of resources within the platform, and social responsibility governance mechanisms (e.g., auditing, credit management, supervision and punishment, and evaluation).

## 4. Conclusion and Future Research

### 4.1. Research Conclusion

A comprehensive analysis of recent studies on smart healthcare systems found that the topic is primarily approached from the macroscopic perspective by considering technology implementation, design principles, and medical applications and that the integrated development of smart healthcare has not been approached from the business model perspective. The theoretical application of this study is summarized as follows. First, this study proposes a business model for smart healthcare information service platforms that applies digital technology to public services and can drive public service supply innovation.

Second, a smart healthcare information service platform is developed from the perspective of value cocreation, a value creation system is constructed through effective interaction with the platform, and value cocreation and value sharing are emphasized as the value proposition of the platform.

Third, from the perspective of business ecology, this study constructs a smart healthcare business ecosystem that can link economic and social considerations and maximize the platform network effect for resource aggregation and utilization to promote the healthy development of the industrial ecosystem.

### 4.2. Future Research

In the context of digital transformation, public service innovation offers great potential. Digital technology fully taps the needs and potential of enterprises, citizens, and nongovernmental organizations and integrates new technology, participants, processes, and channel elements into public service innovation [26]. In addition, there are some limitations and challenges, such as trust crises and governance mechanisms. Due to the lack of clear boundaries and supervision within the smart healthcare information platform, participants in the smart healthcare service ecosystem, while sharing and using resources, may exhibit destructive behaviors, such as the disclosure and abuse of health data, which deviate from the goals of value cocreation. Therefore, future research can explore the sustainability of the model at the external system level, the corporate social responsibility level, and the platform user value proposition level.

This study only proposed a platform business model to provide a new way of thinking about healthcare service innovation. However, the theoretical mechanisms of the model were not quantitatively investigated. Therefore, its applicability and the sustainability of its impact need to be further demonstrated. As public service innovation in the digital transformation scenario, researchers can collect more material for vertical depth of case analysis to adjust the proposed model, further adapting it to the institutional environment and governance practices of China.

## Figures and Tables

**Figure 1:** Framework of the customer service platform business model.

**Figure 2:** Framework of the data-enabled platform business model.

**Figure 3:** A platform business model of healthcare service information.

**Figure 4:** A platform ecosystem with value cocreation.

**Table 1:** Data sources for the case study.

Type of institution	Interviewee	Type of interview	Field observation	Second-hand data
Policy makers and regulators	ZH Health Administration	One field interview with a person in charge of the relevant department	Field visit to the relevant department	Government web page data and related news reports

Medical institutions	People's Hospital of ZHHTI	Field interviews with three people in charge of relevant departments, several communications via phone calls and social media	Field inspection of the implementation of medical informatization and management of the information service platform	Official website, related reports and internal information
	ZHJD Heath Service Center	One field interview with a person in charge of the relevant department	Field inspection of the degree of network informatization	Official website, related reports and internal information

Research and development (R&D) institutions	R&D Center, School of Pharmacy, SYS University	One field interview with a person in charge	Field visits to research centers and laboratories	Research achievements and news reporting from the institution's official website
	ZH United Laboratories	One field interview with a person in charge of the R & D department	Field visits to R & D base, firm headquarters, and exhibition center	News reporting from the institution's official website, industry development reports, and annual reports

Suppliers	ZHHJ Medical Service Management Co., Ltd	One field interview with a marketing manager	Field visit to the business department of the firm	News reporting about the firm, and internal information
	ZHWQ Pharmaceutical Co., Ltd	One field interview with a retail store manager	Field visit to the retail store	Firm's internal reports, annual reports, and official website
	HJ Medical Equipment Co., Ltd	One field interview with a marketing manager	Field visit to the firm's headquarters	Firm's internal reports, annual reports, and official website

**Table 2:** Stakeholders and their interests in a smart healthcare ecosystem.

Stakeholder	Components	Interest	Platform functions
Users	Individuals	Receive healthcare services and access healthcare information	Focus on user needs and collect user feedback, personalized user needs are the basis for decision-making by various stakeholders.
	Families		
	Organizations		

Supervisors	Policymaking and supervisory departments of the government	Promote and regulate the development of the industry	Acquire and share public information resources to provide medical institutions and health supervisory agencies with operational management data and decision analysis

Professional medical institutions	Large general hospitals	Provide clinical decision support, medical information, knowledge sharing; break space-time barriers to provide users with personalized, whole-process healthcare services	Through the sharing of medical big data, address issues such as information asymmetry, inequitable resource allocation, imbalances between supply and demand, inefficiency, and lack of information, thereby improving medical quality and efficiency
	Community hospitals and seniors care facilities		
	Private hospitals		
	Physical examination centers		

Suppliers	Suppliers of technology, medical equipment, pharmaceuticals, training, and solutions	Through information exchange, keep abreast of market conditions, provide relevant products and services according to market demand information, and seek market opportunities	Integrate information from various stakeholders and provide integrated market demand information based on healthcare activity information

R & D institutions	Research institutions	Research and develop new and advanced technologies through the collection of basic medical data and the monitoring of health big data	Driven by applications, integrate information on the platform, including patient access information, clinical medical research and laboratory data, data from pharmaceutical and life science companies, and health management information generated by smart wearable devices, and share data with other R & D firms
	Pharmaceutical firms		

Capital market	Financial institutions	Acquire information on investment returns in the industry and on investment opportunities	Promote cross-border integration through the platform, actively explore commercialization channels, and attract funds from the capital market
	Commercial insurance companies	Ensure medical quality, control costs and expenses, and reduce insurance claims	Promote cooperation with other stakeholders to improve medical quality and control medical costs

Derivative industries	Relevant firms	Actively participate in the development of the smart healthcare system and cooperate with other stakeholders to explore market opportunities	Facilitate the development of strategic cooperation among various stakeholders and diversify business through the information platform

## Data Availability

We conducted an interview study on the stakeholders of the firm that runs the smart healthcare information service platform. For the institutions interviewed, we collected first-hand data through field research and semistructured interviews and, after the interviews, verified and supplemented the data through online channels such as emails or phone calls; in addition, second-hand data were also obtained for quantitative analysis and verification.
